The article "Efficacy of Concomitant Therapy Versus Triple Therapy in Eradicating Helicobacter pylori Infection: A Retrospective Study" was retracted in 2026. Reasons: concerns about the data; concerns about the methods; concerns about the results or conclusions.

# Efficacy of Concomitant Therapy Versus Triple Therapy in Eradicating Helicobacter pylori Infection: A Retrospective Study

**DOI:** 10.7759/cureus.87322

**Published:** 2025-07-05

**Authors:** Muhammad Umair Mazhar, Hafiz Muhammad Ahmad Anees, Samana Mukhtar, Humna Irshad, Ayman Irshad, Abdul Moizz, Abdul Eizad Asif, Hassan Durrani, Haiqa Asif, Hannan Hashmat, Muhammad Khizer Azeem

**Affiliations:** 1 Stroke Medicine, University Hospital Coventry and Warwickshire NHS Trust, Coventry, GBR; 2 Internal Medicine, Allama Iqbal Medical College, Lahore, PAK; 3 Internal Medicine, Hayat Memorial Teaching Hospital, Lahore, PAK; 4 Internal Medicine, Kishwar Fazal Teaching Hospital, Lahore, PAK; 5 Internal Medicine, Shalamar Medical and Dental College, Lahore, PAK; 6 Internal Medicine, Rahbar Medical and Dental College, Lahore, PAK; 7 Internal Medicine, Rashid Latif Medical and Dental College, Lahore, PAK; 8 Internal Medicine, Rawalpindi Medical University, Rawalpindi, PAK

**Keywords:** concomitant, efficacy, eradication, helicobacter pylori, infection, therapy, triple

## Abstract

Background

*Helicobacter pylori*is a widespread bacterial infection that is often linked to significant health and economic burdens in affected populations. The rise of antibiotic resistance has reduced the effectiveness of standard triple therapy (TT), highlighting the need for alternative treatment strategies, especially in resource-constrained countries like Pakistan, where comparative research on different *H. pylori* treatment regimens remains limited. This study aims to compare the efficacy of concomitant therapy (CT) versus TT in the eradication of *H. pylori* infection.

Methods

This retrospective study was conducted over a 12-month period (July 2021 to July 2022) in the medicine and gastroenterology departments of Jinnah Hospital, Lahore, Pakistan. A total of 296 patients diagnosed with *H. pylori* infection via the urea breath test were enrolled using consecutive sampling, following predefined inclusion and exclusion criteria. Patients were divided into two groups of 148 each: Group A received CT (esomeprazole, amoxicillin, clarithromycin, and metronidazole), and Group B received standard TT (esomeprazole, amoxicillin, and clarithromycin). Data were analyzed using IBM SPSS Statistics for Windows, Version 25.0 (Released 2017; IBM Corp., Armonk, NY, USA), applying independent samples t-tests, chi-square tests, and logistic regression analysis. A p-value of less than 0.05 was considered statistically significant.

Results

Among the 296 patients, the overall *H. pylori* eradication rate was 82.09%. The eradication rate was significantly higher in the CT group (91.90%) compared to the TT group (72.29%) (p = 0.008). In the CT group, age (OR: 1.57; 95% CI: 1.25-1.98; p = 0.03) and duration of symptoms (OR: 1.42; 95% CI: 1.10-1.77; p = 0.02) were significant predictors of successful eradication, while gender (OR: 1.10; 95% CI: 1.01-1.32; p = 0.06) was not. In the TT group, age (OR: 1.22; 95% CI: 1.05-1.51; p = 0.06), gender (OR: 1.01; 95% CI: 0.71-1.47; p = 0.07), and duration of symptoms (OR: 1.26; 95% CI: 1.17-1.60; p = 0.09) were not significant predictors of eradication.

Conclusions

This study suggests that CT is more effective than TT in eradicating *H. pylori* infection. In the CT group, being younger than 45 years and having symptoms for less than six months were significant predictors of treatment success. These findings provide valuable insights into optimal treatment strategies for *H. pylori* in resource-limited settings and emphasize the need for further research to establish effective eradication protocols.

## Introduction

*Helicobacter pylori *infection is one of the most prevalent bacterial infections globally, affecting approximately 50% of the world’s population. Its clinical manifestations range from asymptomatic cases to nonspecific symptoms such as abdominal pain, a burning sensation, bloating, nausea, vomiting, and loss of appetite [1]. The bacterium colonizes the gastric mucosa, and if left untreated, can increase the risk of developing peptic ulcer disease by 10-20% and gastric cancer by 1-2%. Less commonly, *H. pylori *infection can also lead to gastric mucosa-associated lymphoid tissue lymphoma [1,2].

Transmission is primarily linked to poor sanitation and hygiene practices, especially in developing countries [3]. Additional risk factors include low socioeconomic status, overcrowded living conditions, consumption of unpasteurized milk or dairy products, and a family history of infection. Children are particularly vulnerable due to their immature immune systems and increased exposure to contaminated environments. Lifestyle choices, including smoking, alcohol consumption, and unhealthy diets, further contribute to susceptibility [4].

Although improvements in hygiene have significantly reduced *H. pylori *prevalence in developed countries, the infection remains widespread in developing regions, with rates ranging from 30.60% to 82% [2,5,6]. In Pakistan, *H. pylori* infection remains a pressing public health concern, with studies reporting prevalence rates as high as 64.20%, varying by province. Similar trends are observed in other low- and middle-income countries [1,7].

The global economic burden of *H. pylori *infection is substantial. In 2016, healthcare expenditures for conditions such as peptic ulcer disease, gastritis, and duodenitis surpassed $2 billion [8]. This burden is particularly significant in developing countries like Pakistan, where healthcare resources are limited. In addition to its economic impact, *H. pylori *poses a serious health risk, contributing to gastric cancer, one of the leading causes of cancer-related mortality worldwide [1,7,9].

A variety of diagnostic tools are available for *H. pylori* infection, including both invasive and noninvasive tests. Invasive methods involve endoscopy with biopsy, while noninvasive options include the urea breath test (UBT), stool antigen test, and serological testing [10]. Standard treatment traditionally involves triple therapy (TT), which includes a proton pump inhibitor (PPI) along with two antibiotics, typically clarithromycin and amoxicillin [4,11].

However, rising antibiotic resistance has reduced the effectiveness of TT in many regions. Studies have shown clarithromycin resistance rates exceeding 50% in some cases [12,13]. To address this, quadruple therapies, either bismuth-based or nonbismuth-based, have been introduced. One such regimen is concomitant therapy (CT), which combines a PPI with metronidazole, clarithromycin, and amoxicillin [14-20].

Despite its potential, data comparing the efficacy of CT and TT remain limited, particularly in resource-limited settings like Pakistan [1,2]. In light of growing resistance and the lack of local evidence, further investigation into the efficacy of CT is warranted.

This study aims to compare the eradication rates of CT versus TT for *H. pylori *infection in a Pakistani population. The findings will help fill an important research gap, providing clinicians and policymakers with evidence-based guidance. Ultimately, this work will support the development of more effective treatment strategies for *H. pylori* infection, with the goal of reducing the burden of gastrointestinal disease and gastric cancer in Pakistan and other developing countries.

## Materials and methods

Study design and study population

This retrospective study was conducted at the Departments of Medicine and Gastroenterology, Jinnah Hospital, Lahore, Pakistan, over a 12-month period from July 2021 to July 2022. A total of 296 patients diagnosed with *H. pylori* infection were enrolled through consecutive sampling, based on predefined inclusion and exclusion criteria. The sample size was calculated using the OpenEpi sample size calculator, referencing a 22% prevalence of *H. pylori* infection in Pakistan as reported by Shah et al. The calculation was based on a 95% CI and a 5% margin of error, with an effect size of 0.528 [1]. Ethical approval was obtained from the relevant institutional review board prior to the commencement of the study.

Inclusion and exclusion criteria

The study included adult patients (aged 18 years or older) of both genders who had a confirmed diagnosis of *H. pylori* infection via the UBT and complete medical documentation. This included past medical and surgical histories, treatment with first-line triple or CT, and complete follow-up data. Patients were excluded if they were under 18 years of age, had severe comorbidities (cardiovascular, respiratory, endocrine, renal, hematological, or hepatic disorders), had previously undergone *H. pylori* eradication therapy or gastric surgery, or had known allergies to any of the antibiotics used in the study. Additional exclusion criteria included pregnancy or lactation, alcohol or substance abuse, use of antibiotics, PPIs, corticosteroids, or NSAIDs within the past four weeks, presence of autoimmune disorders, malignancies, or recent surgeries (within the past three months), as well as noncompliance with therapy or loss to follow-up. These criteria were applied to minimize potential confounding factors affecting treatment outcomes.

Diagnosis of *H. pylori* infection

*H. pylori* infection was diagnosed using a noninvasive UBT. Patients were advised to discontinue PPIs for at least two weeks before testing and were confirmed to have not taken antibiotics for at least four weeks prior. Eradication was assessed using the same test, performed at least four weeks after completion of therapy. A positive result on the UBT indicated treatment failure, whereas a negative result was considered successful eradication of *H. pylori*.

Treatment regimens

Patients were divided into two groups of 148 each. Group A received CT, consisting of esomeprazole 40 mg twice daily, amoxicillin 1 g twice daily, clarithromycin 500 mg twice daily, and metronidazole 500 mg twice daily for 14 days. Group B was treated with TT, comprising esomeprazole 40 mg twice daily, amoxicillin 1 g twice daily, and clarithromycin 500 mg twice daily, also for 14 days. Patients were informed about potential side effects, including a metallic taste, diarrhea, abdominal pain, nausea, and vomiting. Weekly follow-ups were conducted to assess adherence, monitor for adverse events, and evaluate symptom relief. Compliance was defined as taking 100% of the prescribed medications.

Data collection tool

Data were collected from patient medical records using a self-designed pro forma consisting of two sections. The first section recorded demographic information such as age (categorized as below 45 years or 45 years and above), gender, duration of symptoms (less than six months or six months and above), medical history, and physical examination findings. The second section focused on diagnostic test results.

Data analysis

Data analysis was performed using IBM SPSS Statistics for Windows, Version 25.0 (Released 2017; IBM Corp., Armonk, NY, USA). Categorical variables were summarized as frequencies and percentages, while continuous variables were expressed as mean ± SD. An independent samples t-test was used to compare quantitative variables between the two groups. The chi-square test was used for qualitative comparisons. Univariate analysis using the chi-square test assessed the association of variables such as age, gender, and symptom duration with treatment outcomes. Multivariate binary logistic regression was then applied to calculate ORs and 95% CIs, using *H. pylori* eradication as the dependent variable and the aforementioned factors as independent variables. A p-value less than 0.05 was considered statistically significant.

## Results

Out of 296 patients, 243 (82.09%) achieved successful eradication of *H. pylori *infection, while 53 patients (17.91%) did not respond to the treatment they received. The mean age of the study population was 47.60 years, with an SD of ±11.34 years.

Table 1 presents the demographic and clinical characteristics of the study population. It also shows a statistically significant difference in eradication rates between the two treatment groups - CT and TT - with a p-value of 0.008. However, there were no statistically significant differences between the groups regarding age distribution, gender, or duration of symptoms (p > 0.05).

**Table 1:** Analysis of demographic and clinical characteristics of the study population In the second-to-last column, test statistic values marked with an asterisk (^*^) represent results from the independent t-test, while values marked with a plus sign (^+^) correspond to the chi-square test. Similarly, in the last column, p-values marked with an asterisk (^*^) are from the independent t-test, and those marked with a plus sign (^+^) are from the chi-square test. CT, concomitant therapy; TT, triple therapy

Variables with *Helicobacter pylori*infection (n = 296)		Expression of variables	Various therapies applied for *H. pylori*treatment		Chi-square test/independent t-test	
					Test statistics	
			CT group (n = 148; 50%)	TT group (n = 148; 50%)	χ² value for chi-square test/t-value for independent test	p-values
Age (years) (means ± SD)		47.60 ± 11.34	47.08 ± 12.45	47.88 ± 12.65	0.26^*^	0.62^*^
Age groups	Less than 45 years, n (%)	138 (46.62)	78 (52.70)	60 (40.54)	4.71^+^	0.54^+^
	45 years or above, n (%)	158 (53.38)	70 (47.30)	88 (59.46)		
Gender	Male, n (%)	126 (42.56)	62 (41.89)	64 (43.24)	0.40^+^	0.48^+^
	Female, n (%)	170 (57.44)	86 (58.11)	84 (56.76)		
Duration of symptoms	Less than six months, n (%)	142 (47.97)	70 (47.29)	72 (48.64)	0.80^+^	0.78^+^
	Six months or above, n (%)	154 (52.03)	78 (52.71)	76 (51.36)		
Eradication of infection	Yes, n (%)	243 (82.09)	136 (91.90)	107 (72.29)	18.37^+^	0.008^+^
	No, n (%)	53 (17.91)	12 (8.10)	41 (27.71)		

Table 2 shows that the frequency of successful *H. pylori* eradication was higher among patients treated with CT compared to those who received TT. Additionally, it highlights that variations in age group and duration of symptoms had a statistically significant impact on eradication outcomes in the CT group, whereas gender did not show a significant effect. Although similar trends were observed in the TT group - with age, gender, and symptom duration influencing eradication rates - these associations were not statistically significant.

**Table 2:** Crosstabulation of H. pylori infection eradication with variables based on treatment in the study population CT, concomitant therapy; TT, triple therapy

Therapies applied for the eradication of the *Helicobacter pylori*infection	Expression of variables			Eradication of *H. pylori*infection		Chi-square test (test statistics)	
				Group with successful eradication of *H. pylori*infection	Group without eradication of *H. pylori*infection	χ² value for chi-square test	p-values
CT group (n = 148)	Age groups	Less than 45 years, n (%)	78 (52.70)	74 (94.87)	4 (5.13)	2.35	0.03
		45 years or above, n (%)	70 (47.30)	62 (88.57)	8 (11.43)		
	Gender	Male, n (%)	62 (41.89)	58 (93.55)	4 (6.45)	0.35	0.06
		Female, n (%)	86 (58.11)	78 (90.70)	8 (9.30)		
	Duration of symptoms	Less than six months, n (%)	70 (47.29)	67 (95.71)	3 (4.29)	4.24	0.02
		Six months or above, n (%)	78 (52.71)	69 (88.46)	9 (11.54)		
TT group (n = 148)	Age groups	Less than 45 years, n (%)	60 (40.54)	45 (75.00)	15 (25.00)	0.34	0.06
		45 years or above, n (%)	88 (59.46)	62 (70.46)	26 (29.54)		
	Gender	Male, n (%)	64 (43.24)	48 (75.00)	16 (25.00)	0.38	0.07
		Female, n (%)	84 (56.76)	59 (70.24)	25 (29.76)		
	Duration of symptoms	Less than six months, n (%)	72 (48.64)	53 (73.61)	19 (26.39)	0.40	0.09
		Six months or above, n (%)	76 (51.36)	54 (71.06)	22 (28.96)		

ORs and 95% CIs were calculated to assess the association of patient variables with successful *H. pylori* eradication in each treatment group. In the CT group, both age (OR: 1.57; 95% CI: 1.25-1.98; p = 0.03) and duration of symptoms (OR: 1.42; 95% CI: 1.10-1.77; p = 0.02) were significantly associated with successful eradication. Gender (OR: 1.10; 95% CI: 1.01-1.32; p = 0.06) did not show a statistically significant association. These findings suggest that younger age and shorter symptom duration may enhance the effectiveness of CT.

In contrast, no statistically significant associations were found in the TT group. Age (OR: 1.22; 95% CI: 1.05-1.51; p = 0.06), gender (OR: 1.01; 95% CI: 0.71-1.47; p = 0.07), and duration of symptoms (OR: 1.26; 95% CI: 1.17-1.60; p = 0.09) were not predictive of treatment success, indicating limited influence of these variables on TT efficacy.

## Discussion

*H. pylori *is a widespread bacterial infection affecting nearly half of the global population. If left untreated, it can lead to severe gastrointestinal complications, including peptic ulcer disease and a heightened risk of gastric cancer. Despite the availability of multiple treatment options, the increasing rate of antibiotic resistance remains a major obstacle to successful eradication [1,4]. Therefore, assessing the efficacy of alternative regimens is crucial, especially in resource-limited settings. The present study provides valuable insights by comparing the effectiveness of CT and TT while also identifying key predictors of treatment success.

Among the 296 patients included in the study, the overall eradication rate was 82.09%, with 243 patients achieving successful clearance of *H. pylori*. A total of 53 patients (17.91%) failed to respond to their prescribed treatment. This eradication rate aligns with previous research, such as one study reporting a similar frequency of 84.30% [2]. However, other regions have reported lower rates; for instance, a study from Bahrain documented an eradication rate of only 69.90% [12]. Variations in outcomes may be attributed to differences in antibiotic resistance patterns, choice of treatment regimens, and population demographics. These discrepancies underscore the importance of developing context-specific strategies for the eradication of *H. pylori*.

The eradication rates differed significantly between the two treatment groups. Patients who received CT had a substantially higher eradication rate (91.90%) compared to those on TT, who achieved a rate of 72.29%. This finding is consistent with a growing body of literature supporting the superiority of CT. For instance, a study from Greece reported eradication rates of 93.30% for CT and 75.80% for TT [16]. Similarly, research from Spain found CT to be more effective (84.80%) than TT (65.70%) [17]. A meta-analysis of 23 randomized controlled trials reinforced these findings, demonstrating that CT is consistently associated with higher eradication rates [18]. Additional studies from South Korea and a 16-center prospective investigation also reported higher success rates with CT, at 93.40% and 93.80%, respectively, compared to TT [19,20]. These results collectively validate the global effectiveness of CT in *H. pylori* eradication.

Regarding clinical predictors, age under 45 years and symptom duration of less than six months were significant determinants of successful eradication in the CT group. Although eradication rates were higher among males, gender was not a statistically significant factor. In the TT group, the same demographic and clinical trends were observed; however, none of these factors reached statistical significance. Similar associations have been reported in previous studies [2,21]. Younger patients may benefit from stronger immune responses, fewer comorbidities, and higher adherence to treatment. Likewise, a shorter duration of symptoms might reflect less entrenched disease, which may respond more favorably to antibiotics [1,16-20].

The superior performance of CT can be attributed to its use of multiple antibiotics with distinct mechanisms of action, which helps limit the impact of antibiotic resistance and enhances overall treatment efficacy. This makes CT particularly valuable in areas with high levels of resistance [14-19]. To effectively combat resistance, future strategies should consider incorporating bismuth-based quadruple therapies, individualized regimens guided by susceptibility testing, and adjunctive nonantibiotic therapies such as probiotics. A comprehensive and tailored approach is vital for optimizing treatment outcomes [20,21].

This study holds significant implications, particularly for Pakistan and neighboring regions, as it suggests that CT may be a more effective treatment option for *H. pylori *infection compared to TT. These findings could guide clinicians in optimizing patient outcomes through evidence-based decision-making. Despite the emerging evidence supporting newer regimens, the use of TT remains more common in Pakistan, primarily due to limited data on alternative treatments for *H. pylori *infection [1,2,4]. To improve management of this infection in the region, policy changes are warranted. These should include updated treatment guidelines recommending more effective regimens, the implementation of antibiotic stewardship programs, cost-effectiveness evaluations, and assessments of the healthcare burden associated with persistent infection. Such measures would support more effective treatment strategies, help curb antibiotic resistance, and reduce the overall economic impact.

In addition to its clinical relevance, this study has several limitations. Its retrospective design, single-center setting, and exclusion of patients with severe comorbidities may limit the generalizability of the results. Furthermore, antibiotic resistance patterns were not assessed, which may influence treatment efficacy. Future research should explore the effectiveness of CT across diverse populations and evaluate how antibiotic resistance affects treatment outcomes. Prospective, multicenter studies would offer broader and more robust evidence to validate these findings. Moreover, investigating specific patient subgroups, such as older adults and individuals with comorbid conditions, could help refine treatment strategies and support more personalized care.

## Conclusions

This study suggests that incorporating metronidazole into the standard TT regimen significantly enhances treatment outcomes in *H. pylori*infection. CT demonstrated a notably higher eradication rate compared to traditional TT, particularly among patients younger than 45 years and those with symptoms of less than six months’ duration. Gender did not significantly influence outcomes. Although similar demographic patterns were observed in the TT group, they did not reach statistical significance.

Given its retrospective nature, further prospective studies are warranted to confirm these findings. If validated, this evidence could support the integration of CT into routine clinical practice, especially in resource-limited settings. Doing so may not only improve individual patient outcomes but also help reduce the broader economic and healthcare burden posed by persistent *H. pylori* infections.

## References

[1] Shah SR, Almugadam BS, Hussain A, Ahmad T, Ahmed S, Sadiqui S (2021). Epidemiology and risk factors of Helicobacter pylori infection in Timergara city of Pakistan: a cross-sectional study. Clin Epidemiol Glob Health.

[2] Butt AM, Sarwar S, Nadeem MA (2021). Concomitant therapy versus triple therapy: efficacy in H. pylori eradication and predictors of treatment failure. J Coll Physicians Surg Pak.

[3] Burucoa C, Axon A (2017). Epidemiology of Helicobacter pylori infection. Helicobacter.

[4] Amil J, Sajjad S, Khan RA, Majeed S, Ahmed K, Masood MA (2024). Comparison of therapeutic outcomes: two triple-therapy approaches for H. pylori eradication in gastric ulcer disease: two triple-therapy for H. pylori eradication. Pakistan J Health Sci.

[5] Li Y, Choi H, Leung K, Jiang F, Graham DY, Leung WK (2023). Global prevalence of Helicobacter pylori infection between 1980 and 2022: a systematic review and meta-analysis. Lancet Gastroenterol Hepatol.

[6] Yuan C, Adeloye D, Luk TT (20221). The global prevalence of and factors associated with Helicobacter pylori infection in children: a systematic review and meta-analysis. Lancet Child Adolesc Health.

[7] Mujtaba MA, Khan HS, Azhar R, Zulfiqar A, Bukhari SH, Yousaf A (2025). Frequency of Helicobacter pylori infections and its association with immune thrombocytopenia in patients presenting with dyspepsia in tertiary care setting, Islamabad. Life Sci.

[8] Shah S, Hubscher E, Pelletier C, Jacob R, Vinals L, Yadlapati R (2022). Helicobacter pylori infection treatment in the United States: clinical consequences and costs of eradication treatment failure. Expert Rev Gastroenterol Hepatol.

[9] Sardar M, Kumar D, Aakash F (2023). Prevalence and etiology of Helicobacter pylori infection in dyspepsia patients: a hospital-based cross-sectional study. Ann Med Surg (Lond).

[10] Kotilea K, Bontems P, Touati E (2019). Epidemiology, diagnosis and risk factors of Helicobacter pylori infection. Adv Exp Med Biol.

[11] Alawainati M, Ali MM, AlShaalan M, Hasan HI, Jasim QM, Almusawi S (2025). Helicobacter pylori in Bahrain: a comprehensive study of patient characteristics, treatment approaches, and cure rates. Cureus.

[12] Barakat A, Althahabi R, Aljazaf H (2025). The efficacy of quadruple therapy versus triple therapy in Helicobacter pylori eradication. Cureus.

[13] Hong TC, El-Omar EM, Kuo YT (20241). Primary antibiotic resistance of Helicobacter pylori in the Asia-Pacific region between 1990 and 2022: an updated systematic review and meta-analysis. Lancet Gastroenterol Hepatol.

[14] Chey WD, Howden CW, Moss SF, Morgan DR, Greer KB, Grover S, Shah SC (2024). ACG clinical guideline: treatment of Helicobacter pylori infection. Am J Gastroenterol.

[15] Jung HK, Kang SJ, Lee YC (2021). Evidence-based guidelines for the treatment of Helicobacter pylori infection in Korea 2020. Gut Liver.

[16] Georgopoulos S, Papastergiou V, Xirouchakis E (2013). Nonbismuth quadruple "concomitant" therapy versus standard triple therapy, both of the duration of 10 days, for first-line H. pylori eradication: a randomized trial. J Clin Gastroenterol.

[17] Campillo A, Ostiz M, Amorena E, Kutz M, La Iglesia M (2016). Quadruple concomitant non-bismuth therapy vs. classical triple therapy as first line therapy for Helicobacter pylori infection. Med Clin.

[18] Chen MJ, Chen CC, Chen YN (2018). Systematic review with meta-analysis: concomitant therapy vs. triple therapy for the first-line treatment of Helicobacter pylori infection. Am J Gastroenterol.

[19] Molina-Infante J, Lucendo AJ, Angueira T (2015). Optimised empiric triple and concomitant therapy for Helicobacter pylori eradication in clinical practice: the OPTRICON study. Aliment Pharmacol Ther.

[20] Kim SY, Lee SW, Choe JW (2017). Helicobacter pylori eradication rates of concomitant and sequential therapies in Korea. Helicobacter.

[21] Yan TL, Gao JG, Wang JH, Chen D, Lu C, Xu CF (2020). Current status of Helicobacter pylori eradication and risk factors for eradication failure. World J Gastroenterol.

